The article "Diagnostic Efficacy and Clinical Value of Ultrasonography in Difficult Airway Assessment: Based on a Prospective Cohort Study" was published in 2022. Journal: Contrast Media Mol Imaging.

# Diagnostic Efficacy and Clinical Value of Ultrasonography in Difficult Airway Assessment: Based on a Prospective Cohort Study

**DOI:** 10.1155/2022/4706438

**Published:** 2022-08-24

**Authors:** Huihui Wu, Hong Wang

**Affiliations:** Department of Anesthesiology, Shanghai General Hospital, Shanghai 201600, China

## Abstract

**Objective:**

A case-control study was conducted to explore the diagnostic efficacy and clinical value of ultrasound in difficult airway assessment.

**Methods:**

A total of 220 patients undergoing elective surgery under general anesthesia were prospectively enrolled in our hospital from April 2018 to April 2021. General data were collected one day before operation, including sex, age, height, weight, body mass index (BMI), modified Mallampati test (MMT), inter-incisor distance (IID) and thyromental distance (TMD), the upper lip bite test (ULBT), and thyromental height (TMH). DSH, DSE, DSV, HMD, and tongue width and thickness were measured by ultrasound in the supine position before anesthesia induction on the day of operation. The above data were measured by the same anesthesiologist. After anesthesia, the patients were exposed to laryngoscope by the same senior doctor who did not participate in the data analysis, and the Cormack–Lehane (CL) grade was recorded and endotracheal intubation was completed. The relationship between DSE, DSH, DSV, HMD, and tongue width and thickness and laryngoscope exposure difficulty and tracheal intubation difficulty was analyzed. The critical value of each index for predicting laryngoscope exposure difficulty and tracheal intubation difficulty was obtained by the receiver operating characteristic curve (ROC) and Jordan index. According to the critical value, the accuracy, sensitivity, specificity, positive predictive value, and negative predictive value of each index were calculated.

**Results:**

On comparing the general conditions of the four groups, this study prospectively included 220 patients undergoing elective surgery under general anesthesia for tracheal intubation in our hospital from April 2018 to April 2021, of which 8 cases were excluded from the study because of loss of incisors, 5 cases were excluded from the study due to unclear development of the anterior vocal cords under ultrasound, 7 cases were excluded from the study, and finally 200 patients were included in the study, including 104 males and 96 females. Among the 200 patients, difficult laryngoscope exposure was found in 26 cases (13.00%) and difficult tracheal intubation in 17 cases (8.50%). Tracheal intubation was performed in 17 patients with a visual laryngoscope and light rod, respectively. The weight and BMI of patients in the DL group were higher than in the NDL group, and the difference was statistically significant (*P* < 0.05); the weight and BMI of patients in the DI group were higher than in the NDI group, and the difference was statistically significant (*P* < 0.05); there was no significant difference in sex, age, and height between the DL group and the NDL group and the DI group and the NDI group (*P* > 0.05). Compared with the NDL group, IID, TMD, and TMH in the DL group were lower, and the difference was statistically significant (*P* < 0.05); there was no significant difference in ULBT (*P* > 0.05). DSE, DSH, and DSV were higher than in the NDL group, and the difference was statistically significant (*P* < 0.05), the HMD was lower than in the NDL group, and the difference was statistically significant (*P* < 0.05);the width and thickness of tongue were higher than in the NDL group, and the difference was statistically significant (*P* < 0.05). On comparing the DI NDI groups, the IID, TMD, and TMH in group DI were lower than in group NDI, and the difference was statistically significant (*P* < 0.05), but there was no significant difference in ULBT (*P* > 0.05); DSE, DSH, and DSV were higher than in the NDI group, and the difference was statistically significant (*P* < 0.05); the HMD was lower than in the NDI group, and the difference was statistically significant (*P* < 0.05); the width and thickness of tongue were higher than in the NDL group, and the difference was statistically significant (*P* < 0.05). The AUC of BMI, TMH, DSE, DSV, HMD, and tongue width and thickness all ranged from 0.70 to 0.9. Laryngoscope exposure difficulty diagnostic value was medium. The AUC of TMD, MMT, ULBT, IID, and DSH ranged from 0.5 to 0.7. The diagnostic value of laryngoscope exposure difficulty was low. According to the ROC curve, the AUC value of HMD, DSE, and tongue thickness in ultrasonic indicators was higher than that of traditional indicators and the AUC value of TMH was the highest in traditional indicators. When the HMD cutoff value was 5.29 cm; the accuracy, sensitivity, specificity, PPV, and NPV were 73.6%, 96.7%, 71.6%, 31.8%, and 97.4%, respectively. Compared with tongue width, tongue thickness has a better predictive performance. The accuracy of DSH, DSV, DSE, and tongue width and thickness in predicting difficult laryngoscope exposure was lower than HMD and the difference was statistically significant (*P* < 0.05). The patients in the DI and NDI groups indicated that the AUC of ULBT, TMD, and IID was between 0.5 and 0.7, the diagnostic values of BMI, MMT, TMH, DSE, DSH, DSV, HMD, and tongue width and thickness were between 0.7 and0.9, and the diagnostic value for tracheal intubation difficulty was moderate. According to the ROC curve, HMD, DSE, and tongue thickness in ultrasonic indexes were higher compared to traditional indexes. Among the traditional indexes, the AUC value of TMH is the largest. In ultrasonic indexes, when the critical value of HMD DSE is 4.85 cm, the AUC value is 0.893, and its accuracy, sensitivity, specificity, PPV, and NPV are 81.6%, 93.8%, 80.6%, 30.2%, and 99.5%, respectively. In ultrasonic indexes, the prediction performance is better, followed by the tongue thickness prediction performance. The accuracy of DSH, DSV, DSE, and tongue width and thickness in predicting difficult tracheal intubation was lower than in HMD, and the difference was statistically significant (*P* < 0.05).

**Conclusion:**

Ultrasonic measurements such as DSH, DSE, DSV, HMD, and tongue width and thickness have predictive value for difficult airway;when the ultrasonic measurement of HMD is ˂5.29 cm, we should pay attention to the difficulty of laryngoscope exposure, and when DSE is ˂4.85 cm, we should watch out for difficult tracheal intubation. In terms of other ultrasound indexes, HMD is more valuable in predicting difficult airway.

## 1. Introduction

It is very important to ensure the patency of the respiratory tract and effective ventilation in perioperative period, and airway management is a clinical skill that anesthesiologists must master [1]. Difficult airway can be assigned into expected difficult airway and unanticipated difficult airway; the former includes a clear history of difficult airway, facial scar, and severe obstructive sleep apnea syndrome. For the expected difficult airway, the focus of clinical treatment is to maintain the patient's spontaneous breathing and avoid the occurrence of emergency airway. Ma et al. indicated in a survey of Chinese anesthesiologists conducted in 2020 that 63.2% of anesthesiology departments had cancelled or delayed operations due to difficult airway, and 13.8% had cases of serious adverse events (patient death or brain injury, etc.) caused by difficult airway [2]. Crosby et al. reviewed the 406 anesthesia-related civil litigation cases recorded by the Canadian Medical Protection Association from 2007 to 2016, and concluded that 11% of the disputes were caused by failure of airway management [3]. The incidence of difficult airway is different in different literature. The incidence of difficult airway in elective surgery is 0.7%–27%, and that in pediatrics is about 3.6% [4]. The incidence of difficult laryngoscope exposure was 6.6%–8.0% [5]. Therefore, difficult airway is still one of the core tasks of safety management in anesthesiology departments.

Difficult airway is mainly assigned into difficult mask ventilation, difficult laryngoscope exposure, and difficult tracheal intubation [6]. In the C-L, grades I and II are easy to intubate, grade III is more difficult to intubate, and grade IV is obviously difficult to intubate. The higher the C-L grade, the more difficult it is to intubate, and the failure rate of intubation increases. Difficult airway management failures account for 30% of anesthesia-related deaths, but if difficult airways can be identified before operation, preparing to deal with difficult airways step by step will significantly improve patient safety and avoid difficult airways turning into unpredictable emergency airways; thus, how anesthesiologists evaluate airways and enhance the ability to identify difficult airways is very important to airway management [7].

At present, the commonly used clinical evaluations of difficult airway indicators are neck circumference, MMT, IID, TMD, SMD, head and neck mobility, and the upper lip occlusion test [8]. These traditional airway assessment indicators are simple and easy to use, but the effect of single use is not satisfactory, Ji et al. pointed out in a meta-analysis including 133 studies. The aggregate sensitivity of the routine airway evaluation index was 0.22–0.67 (the sensitivity of mouth opening was 0.22 and that of the upper lip occlusion test was 0.67) [9]. Another meta-analysis of 177088 people indicated that the area under the ROC curve of the commonly used clinical MMT was only about 0.7, which could not be used as a single index for evaluating difficult laryngoscopy or difficult airway [8]. In addition to the above-mentioned indexes, new methods for predicting difficult airway, such as the TMH, height-to-chin distance ratio (RHTMD), and tongue-chin distance ratio (HMDR) in different positions, have been put forward in recent years [10]. Yanna et al. considered that the sensitivity and specificity of TMH and RHTMD in predicting difficult laryngoscope exposure were higher compared to traditional airway assessment indexes MMT, TMD, and SMD [11]. Rana et al. considered that the tongue-chin distance ratio between the head and neck in the extended position and the head and neck in the neutral position is a reliable predictor of difficult airway in clinics, but there is lack of clinical data support from large samples [12]. Conclusively, there are many evaluation indicators of clinical difficult airway, but there is no single reliable index to predict difficult airway, and our exploration of difficult airway evaluation has not stopped.

Ultrasound is a safe, fast, convenient, real-time, and repeatable imaging technology [13]. In recent years, bedside ultrasound technology has been developed day by day. Ultrasound-guided arteriovenous puncture, peripheral nerve block, epidural puncture, volume management, and other techniques have been widely adopted in clinics, and the perioperative management of anesthesiologists has become more inseparable from bedside ultrasound. Nowadays, ultrasound has been widely adopted in airway management. Some scholars believe that ultrasound can provide visual anatomical information of the upper airway, make up for the lack of bedside examination, and help diagnose difficult airway [14]. Other scholars believe that ultrasonic examination of the thickness of the anterior soft tissue in the neck at the level of the hyoid and thyrohyoid membrane can be adopted to distinguish difficult laryngoscope exposure. A number of studies have indicated that the ultrasonic measurement of the distance from the epiglottis to skin and the thickness of the pre-epiglottic space can better predict the occurrence of difficult laryngoscope exposure [13, 14]. In addition, ultrasonic measurement of tongue thickness, tongue longitudinal cross-sectional area, and tongue volume are also good indicators for predicting difficult laryngoscope exposure. At present, the measurement indexes of ultrasonic evaluation of difficult airway are mainly focused on the anterior cervical soft tissue thickness of the epiglottis, hyoid bone, and vocal cord at different anatomical levels. There are a few studies on the measurement of tongue volume combined with anterior cervical skin and soft tissue thickness to predict difficult laryngoscope exposure [15]. The purpose of this study is to pass an observational diagnostic study. To evaluate the predictive value of the ultrasonic measurement of hyoid to skin (DSH), epiglottis to skin (DSE), anterior commissure of vocal cords to skin (DSV), thyroid isthmus tracheal ring to skin (DST), tongue cross section width, tongue longitudinal section area, and tongue volume to difficult laryngoscope exposure, and compared with traditional airway evaluation indexes, so as to provide a new method for clinical difficult airway evaluation. Based on this, 220 patients who were scheduled to undergo elective surgery under general anesthesia tracheal intubation in our hospital from April 2018 to April 2021 were studied, which is reported as follows.

## 2. Patients and Methods

### 2.1. General Information

This study prospectively included 220 patients undergoing elective surgery under general anesthesia for tracheal intubation in our hospital from April 2018 to April 2021, of which 8 cases were excluded from the study because of loss of incisors, 5 cases were excluded from the study due to unclear development of the anterior vocal cords under ultrasound, 7 cases were excluded from the study, and finally 200 patients were included in the study, including 104 males and 96 females. Among the 200 patients, difficult laryngoscope exposure was found in 26 cases (13.00%), difficult tracheal intubation in 17 cases (8.50%), and tracheal intubation was completed in 17 patients with a visual laryngoscope and light stick, respectively. There was no significant difference in all aspects of the general data of all patients (*P* > 0.05), as indicated in Table 1. This study was permitted by the Medical Ethics Association of our hospital, and all patients signed informed consent:

  Selection criteria were as follows: (1) over 18 years old, regardless of sex; (2) ASA grade I-III; (3) patients undergoing elective surgery under general anesthesia after endotracheal intubation; and (4) the clinical data are complete.
  Exclusion criteria were as follows: (1) patients with mouth opening <2.5 cm; (2) patients with obviously limited cervical mobility; (3) patients with maxillofacial deformities, scars, and huge masses; (4) heart, brain, kidney, and other important organs' dysfunction; (5) patients who need awake intubation; (6) previous neck surgery (such as thyroid surgery); and (7) lack of important data.

### 2.2. Treatment Methods

#### 2.2.1. Preoperative Visit

The general data were collected one day before the preoperative visit, including sex, age, height, weight, BMI, MMT, IID, TMD, ULBT, and TMH.

#### 2.2.2. Preparation before Anesthesia

After entering the room, the patients received routine oxygen inhalation, opened the peripheral veins, and monitored pulse oxygen saturation, electrocardiogram, and upper limb non-invasive blood pressure.

#### 2.2.3. Ultrasonic Measurement

The patient goes to the pillow and lies flat, with his head in the middle and leaning back as far as possible, keeping his mouth closed. DSH, DSE, DSV, HMD, and tongue width and thickness were measured (see Figure 1). All the above data were collected by the same anesthesiologist.

#### 2.2.4. Anesthesia Induction

Anesthesia induction was performed after ultrasonic measurement, and the same induction scheme was adopted in all patients undergoing elective surgery. Sufentanil 0.3–0.5 ug/kg, propofol 2-3 mg/kg, and cis atracurium 0.15 mg/kg were given intravenously after pure oxygen ventilation (5 min).

#### 2.2.5. Anesthesia Intubation

After the muscle relaxation was complete, the glottis was exposed with direct laryngoscope by the same anesthesiologist who did not participate in the analysis of airway evaluation results. C-L grading was recorded: grades I and II were regarded as easy exposure of laryngoscope (grade I was full exposure of the glottis under a laryngoscope, while grade II was only the arytenoid cartilage and posterior glottis exposed by a laryngoscope). Grades III and IV were regarded as laryngoscope exposure difficulty (grade III was only the epiglottis exposed to a laryngoscope, while grade IV was invisible under the laryngoscope) and endotracheal intubation. If the failure of endotracheal intubation was diagnosed as difficult airway after more than three times of laryngoscope exposure, the difficult airway should be dealt with immediately, and other intubation tools (light stick, visual laryngoscope, fiberoptic bronchoscope, etc.) should be used for intubation.

#### 2.2.6. Anesthesia Maintenance

After endotracheal intubation was completed, volume-controlled ventilation mode was used, tidal volume was 6–8 mL/kg, and the respiratory rate was adjusted to maintain PetCO_2_ at 35–45 mmHg. All patients were treated with the same regimen: propofol 4–6 mg/kg/h and remifentanil 0.1–2 ug/kg/min. Muscle relaxants were given intermittently to maintain anesthesia and keep the depth of anesthesia between 40 and 60.

### 2.3. Observation Index

Sex, age, height, weight, BMI, MMT, IID, TMD, ULBT, TMH, DSH, DSE, DSV, HMD, and tongue width and thickness were recorded. The C-L grade and whether intubation was difficult were assessed before intubation.

### 2.4. Statistical Analysis

SPSS23.0 statistical software was adopted to process the data. The measurement data were presented as ($\bar{x}$ ± *s*). The group design *t*-test was adopted for the comparison and the analysis of variance was adopted for the comparison between multiple groups. Dun-net-t test was adopted for comparison with the control group. The counting data were presented in the number of cases and the percentage, *χ*^2^ test was adopted for comparison between groups, and the bilateral test was employed for all statistical tests. The ROC curve of the traditional and ultrasonic measurement indexes were drawn and the AUC value was calculated; the prediction performance of each parameter was analyzed and evaluated. Statistically, the actual value range of AUC value was 0.5–1. The diagnostic value was lower when AUC was 0.5–0.7, moderate when AUC was 0.7–0.9, and higher when AUC >0.9. The Youden index was adopted to determine the best predictive standard value of each parameter and its accuracy, sensitivity, specificity, PPV, NPV were *P* < 0.05. The difference exhibited was statistically significant.

## 3. Results

### 3.1. Comparison of the General Conditions of Patients in the Four Groups

First of all, we compared the general conditions of the four groups of patients. This study prospectively included 220 patients undergoing elective surgery under general anesthesia for tracheal intubation in our hospital from April 2018 to April 2021. Among them, 8 cases were excluded from the study due to loss of incisors, 5 cases were excluded from the study due to unclear development of the anterior cords under ultrasound, 7 cases were excluded from the study, and finally 200 patients were included in the study. There were 104 males and 96 females. Among the 200 patients, difficult laryngoscope exposure was found in 26 cases (13.00%), difficult tracheal intubation in 17 cases (8.50%), and tracheal intubation was completed in 17 patients with a visual laryngoscope and light stick, respectively. The weight and BMI of patients in the DL group were higher compared to the NDL group, and the difference was statistically significant (*P* < 0.05); the weight and BMI of patients in the DI group were higher compared to the NDI group, and the difference was statistically significant (*P* < 0.05); there was no significant difference in sex, age, and height between the DL group and the NDL group, and the DI group and the NDI group (*P* > 0.05). The specific results are indicated in Table 1.

### 3.2. Comparison of the Measurement Indexes among the Four Groups of Patients

We compared the measurement indexes of the four groups. Compared with the NDL group, the IID, TMD, and TMH of the DL group were lower, and the difference was statistically significant (*P* < 0.05); there was no significant difference in ULBT (*P* > 0.05); DSE, DSH, and DSV were higher compared to the NDL group, and the difference was statistically significant (*P* < 0.05); the width and thickness of tongue were higher compared to the NDL group, and the difference was statistically significant (*P* < 0.05). Compared with the NDI group, IID, TMD, and TMH in the DI group were lower compared to the NDI group, and the difference was statistically significant (*P* < 0.05); there was no significant difference in ULBT (*P* > 0.05); DSE, DSH, and DSV were higher compared to the NDI group, and the difference was statistically significant (*P* < 0.05); the width and thickness of tongue were higher compared to the NDI group, and the difference was statistically significant (*P* < 0.05). All the results are indicated in Table 2.

### 3.3. Prediction of the ROC Curve of Difficult Laryngoscope Exposure by Different Indexes

We analyzed the ROC curves for different indicators to predict difficult laryngoscopy exposure. The AUC of BMI, TMH, DSE, DSV, HMD, and tongue width and thickness all ranged from 0.70 to 0.9. Laryngoscope exposure difficulty diagnostic value was medium. The AUC of TMD, MMT, ULBT, IID, and DSH ranged from 0.5 to 0.7. The diagnostic value of laryngoscope exposure difficulty is low. According to the ROC curve, the AUC value of HMD, DSE, and tongue thickness in ultrasonic indicators was higher than that of traditional indicators, and the AUC value of TMH was the highest in traditional indicators. When the HMD cutoff value was 5.29 cm, the accuracy, sensitivity, specificity, PPV, and NPV were 73.6%, 96.7%, 71.6%, 31.8%, and 97.4%, respectively. Compared with tongue width, tongue thickness has a better predictive performance. The accuracy of DSH, DSV, DSE, and tongue width and thickness in predicting difficult laryngoscopy exposure was lower than HMD, and the difference was statistically significant (*P* < 0.05). All results are shown in Figures 2 and 3 and Tables 3 and 4.

### 3.4. ROC Curve Analysis of Difficult Endotracheal Intubation Predicted by Different Indexes

We analyzed the ROC curve of difficult tracheal intubation predicted by different indexes. The patients in the DI and NDI groups indicated that the AUC of ULBT, TMD, and IID was between 0.5 and 0.7, the diagnostic value of BMI, MMT, TMH, DSE, DSH, DSV, HMD, and tongue width and thickness was between 0.7 and 0.9, and the diagnostic value for tracheal intubation difficulty was moderate. According to the ROC curve, HMD, DSE, and tongue thickness in ultrasonic indexes were higher compared to traditional indexes. Among traditional indexes, the AUC value of TMH is the largest. In ultrasonic indexes, when the critical value of HMD is 4.85 cm, the AUC value is 0.893, and its accuracy, sensitivity, specificity, PPV, and NPV are 81.6%, 93.8%, 80.6%, 30.2%, and 99.5%, respectively. In ultrasonic indexes, the prediction performance is better, followed by the tongue thickness prediction performance. The accuracy of DSH, DSV, DSE, and tongue width and thickness in predicting difficult tracheal intubation was lower compared to HMD, and the difference was statistically significant (*P* < 0.05). All the data results are indicated in Figures 4 and 5 and Tables 5 and 6.

## 4. Discussion

Difficult airway usually refers to a clinical condition in which trained anesthesiologists encounter difficulties in mask ventilation or endotracheal intubation [15]. In the process of difficult airway management, there can be complications such as tooth loss and airway injury. Failure to establish artificial airway will lead to serious adverse consequences such as hypoxia, cardiac arrest, brain injury, and even death in a short time [15, 16]. A patients whose risk factors of difficult airway were not found by preoperative evaluation may have emergency airway after anesthesia induction, i.e., “neither intubation nor ventilation” due to unanticipated difficult airway. It even causes serious adverse consequences such as hypoxia, asphyxia, brain injury, or even death. Some scholars have studied 406 forensic records of the Canadian Medical Protection Society from 2006 to 2016. It was found that 11% (*n* = 46) of the cases were associated with airway management failure, of which 56% (*n* = 26) were caused by inadequate airway assessment, and about 2/3 (*n* = 30) led to serious adverse clinical outcomes such as death and permanent brain damage [16]. Thus, it can be noticed that a sound airway assessment is very important for clinical safety and quality assurance.

If the unexpected difficult airway can be identified before operation, the safety of patients will be significantly improved if they are prepared to deal with the difficult airway step by step. At present, there are many methods for predicting difficult airway in clinics. These methods have certain sensitivity and specificity, but the ideal prediction result cannot be achieved using a certain index alone. Several commonly used clinical indicators are often used together to enhance the ability to predict difficult airways. For example, the El-Ganzouri risk scale (EGRI), proposed by AmerGF through observation of difficult airways, includes seven factors: mouth opening, nail-chin distance, modified Markov grade MMT, cervical range of motion, mandibular protrusion ability, body weight, and previous history of difficult airway disease [17]. Iacovazzo et al. through a retrospective analysis of 2747 cases concluded that the EGRI scale has a higher ability to predict difficult airway, but it contains more parameters and the measurement process is tedious, which limits its clinical application [18]. Elbakery et al. believe that the sensitivity and specificity of predicting difficult airway by combining modified Mahalanobis classification, atlantoaxial range of motion, nail-chin distance, and horizontal length of mandible can reach 77.8% and 92.40% accuracy, respectively, which is better than using one of these indexes alone [19]. Some scholars believe that the possible cause of this phenomenon is that the difficult airway itself is caused by a variety of risk factors.

In the past, it has been reported that imaging methods such as CT and MRI can be used to evaluate difficult airway [20]. Although both CT and MRI can provide a clear anatomical structure of the airway, they have the disadvantages of high price, inconvenient operation, radioactivity, and cannot provide dynamic anatomical images of the airway, which limits their clinical application. With the advantages of convenient bedside examination, dynamic image, low cost, and no radiation, ultrasound has a place in perioperative application and is favored by clinicians and anesthesiologists [21]. For example, ultrasound-assisted arterial catheterization, ultrasound-guided regional nerve block and pain management, ultrasound-assisted lumbar puncture anesthesia, ultrasound evaluation of gastric content volume to prevent reflux aspiration, and other techniques have been widely adopted in clinical practice. Meanwhile, ultrasound is more widely adopted in airway management, such as ultrasound-assisted recognition of cricothyroid membrane, ultrasound-assisted prediction of tracheal intubation size, and determination of endotracheal intubation location. Ultrasound can perform immediate and dynamic airway assessment at the bedside and avoid direct contact with patients; perhaps, in this particular scenario, the use of ultrasound is more promising.

Two hundred patients were included in this study, including difficult laryngoscope exposure in 26 cases (13.00%) and difficult tracheal intubation in 17 cases (8.50%). There is a great difference between difficult laryngoscope exposure and difficult intubation, which can be attributed to many factors, such as ethnic differences, head position, and extralaryngeal pressure. The results of this study are similar to those of Andruszkiewicz et al. (11.1%) [22]. What is different from the expected results is that BMI can predict difficult laryngoscope exposure and difficult tracheal intubation, which may be related to population differences and sample size. There is no correlation between age and the occurrence of difficult airway, which is not consistent with the view of Yao and Wang [23].

Among the traditional evaluation indexes, TMH has the best prediction performance, taking the critical value 4.81 cm. TMH was proposed by Etezadi et al. [24]. The patient goes to the pillow and the mouth is closed, and a straight line parallel to the long axis of the body is made through the mental bone and the thyroid cartilage, respectively. THM refers to the distance between the two straight lines. It is found that when TMH <5 cm, laryngoscope exposure is difficult, and the prediction and evaluation of difficult airway is better than TMD and MMT. Panjiar et al. found that when the cutoff value was 5.1 cm, the AUC value was 0.841, and the sensitivity, specificity, PPV, and NPV were 78.18%, 93.94%, 58.90%, and 97.48%, respectively [25]. However, the critical value of Yanna et al. is 4.9 cm, and the result of this study is similar to that of Yanna et al. Although there are differences among the statistical values of each study, TMH is still the best compared with other evaluation indicators, which is consistent with previous studies. Selvi et al. previously reported that TMH has a lower PPV (20.87% PPV when TMH <43.52 mm, PPV is 14.66% when TMH <50 mm) [26]. The reason for the low PPV value is that the thyroid cartilage of men is more prominent, which leads to false positive.

MMT is the most widely adopted in predicting difficult airway. MMT is evaluated and graded according to the degree of glottis peeping when the root of the tongue increases disproportionately. The evaluation method is that when the patient takes the upright sitting position, he should open his mouth as wide as possible and keep his tongue silent as much as possible. Grade I: soft palate, palatopharynx arch, uvula; grade II: soft palate, palatopharynx arch, part of uvula covered by the root of tongue body; grade III: only soft palate; grade IV, only hard palate, no soft palate [25]. Among them, grade I-II intubation is easy, while grade III-IV intubation is difficult. In this study, the sensitivity, specificity, PPV, and NPV of predicting difficult intubation were 72.7%, 33.5%, 9.0%, and 93.2%, respectively, which was similar to that of Panjiar et al. Meta-analysis results indicated that MMT independently predicted difficult laryngoscope exposure or difficult intubation was not valuable, but it could be a part of a multivariate prediction model. TMD refers to the distance from the lower margin of the mandible to the thyroid cartilage notch when the neck is fully extended, and it is also a simple and convenient evaluation index commonly used in clinics. Adult patients take 6.5 cm as the dividing point; 6.0 cm < TMD < 6.5 cm, if there are no other anatomical abnormalities, it is generally feasible to endoscope and intubation, while TMD <6 cm is difficult to peep into the larynx.

In this study, the accuracy of TMD in predicting difficult laryngoscope exposure is 80.4%, but its sensitivity is 39.7%, which is similar to the accuracy and NPV of Panjiar et al. studies. ULBT can evaluate the range of mandibular movement and the structure of teeth. The grading standard is grade I: the lower incisor can bite above the red edge of the upper lip; grade II: the lower incisor can bite below the red edge of the upper lip; grade III the lower incisor cannot bite the upper lip; and grade III indicates that it is difficult to intubate. In this study, the sensitivity, specificity, PPV, NPV, and accuracy of ULBT in predicting laryngoscope were similar to those of HonarmandA and other people[27]. Xu and Zuo Leila made the same comparison, but the results were different [28]. The recognition rates of both were lower, and the score of ULBT (0.60 [95%CI:0.57–0.63]) was lower compared to Mallampati (0.66 [95%CI:0.63–0.69]). This study is consistent with Eberhart's research.

Ultrasound has been proved to be meaningful in predicting difficult airways, but at present, there are many measurement indexes, and there is still no consensus and standard on which parameter is the best [28, 29]. The upper respiratory tract is formed by two curves, namely the oropharynx curve and the pharynx-glottis-trachea curve. Laryngoscope fully exposed glottis requires that the two curves must be aligned with the visual axis. The increase of DSE may increase the upward concavity of the oropharyngeal curve, make the visual axis deviate from the glottis during direct laryngoscope examination, and narrow the line of sight, thus affecting the glottis exposure. In this experiment, when the cutoff value of DSE is 1.78 cm, the accuracy, sensitivity, specificity, PPV, and NPV were 73.6%, 96.7%, 71.6%, 31.8%, and 97.4%, respectively. Compared with other ultrasonic indexes, the diagnostic performance is the highest. The results of this study are consistent with those of Zheng et al. [29] and Nazir and Mehta [30], and have roughly the same cutoff point. Zheng et al. conducted a study in the Han population, including 203 patients. The results indicated that the critical point of laryngoscope for DSE diagnosis was 1.78 cm, with a sensitivity of 100.0% and a specificity of 66.3%. However, the cutoff points of DSE vary greatly among many research results. One preliminary experiment indicated that the cutoff value of DSE was 2.8 cm, while another study suggested that the cutoff point of DSE was 2.75 cm, with a sensitivity of 64.7% and a specificity of 77.1%. The differences in the results of the study may be related to the differences in the researchers' experience in ultrasound scanning and ultrasound use, the differences in the operators' experience in laryngoscopy, and whether external laryngeal pressure is pressurized or not. In addition, differences among different ethnic groups will also affect the results of the study, and it is pointed out that the difference in the observation results is due to the difference in fat distribution between different races.

According to the ROC curve, the critical value of DSH for predicting laryngeal snooping difficulty is 0.89 cm, the sensitivity is 71.6%, the specificity is 48.3%, the preciseness is 91.7%, and the accuracy is 51.8%. In the study of other scholars. DSH predicted that the average value of difficult laryngoscopy was 0.7 cm, the sensitivity of the test was 75%, the specificity was 54%, the specificity of NPV was 98.1%, and the diagnostic accuracy was only 55%. This study is similar to its results. However, other scholars indicated that DSH had a higher correlation with difficult laryngoscope exposure than other ultrasonic indexes, and the AUC value for predicting difficult laryngoscope exposure was 0.66 (95%CI: 0.547–0.772), which was higher compared to DSE. The critical value of DSV for predicting laryngoscope was 0.745 cm, and the sensitivity, specificity, PPV, NPV, and accuracy were 66.0%, 66.3%, 23.0%, 92.7%, and 66.3%, respectively. Some studies have found that difficult laryngoscopy is related to the thickness of the soft tissue at the level of the vocal cord. Zheng et al. studies also support that DSV can predict difficult intubation, but there is no significant difference in soft tissue thickness between laryngoscope exposure difficulty group and non-laryngoscope exposure difficulty group in the preliminary test of other scholars.

The tongue is a muscular organ in the oral cavity, and it along with its adjacent tissue structures plays an important role in airway evaluation. Hypertrophy of the tongue may affect laryngoscope exposure. Statistical analysis results indicate that it can predict difficult airway. When the cutoff value 5.56 cm is taken, the sensitivity, specificity, accuracy, and AUC value of predicting difficult laryngoscope exposure are 75.6%, 68.4%, 69.4%, and 0.776, respectively. Some studies have found that >6.1 cm is an independent risk factor for predicting difficult airway, with a sensitivity of 0.75 (95%CI: 0.60–0.86) and a specificity of 0.72 (95%CI: 0.70–0.74). It is pointed out that ultrasonic measurement is a more accurate index to predict the difficulty of laryngoscope examination in pregnant women than MMT and IID. When >5.865 cm, the area under the exposure curve of difficult laryngoscope is 0.93 (95%CI: 0.88–0.98), and the sensitivity and specificity are 85% and 91%, respectively. The results of Yadav et al. also believe that it can predict difficult laryngoscopy, and its sensitivity and specificity are 71% and 72%, respectively [31]. At present, there are only a few experiments conducted to study the predictive value of HMD on laryngoscope exposure and intubation. The results of this experimental study indicate that the ultrasonic measurement of HMD >4.36 cm may be a predictor of laryngoscope exposure difficulty, with a sensitivity of 88.6%, a specificity of 55.7%, a specificity of 55.7%, a NPV of 23.6%, an AUC value of 0.738, and its predictive ability needs to be further studied.

This study has some limitations: the sample size of this study is small, it belongs to a single-center study, and there is a certain deviation. There are patients' own factors and other confounding factors that may interfere with the accuracy of this study. In future research, we will carry out multicenter, large sample prospective studies, or we can draw more valuable conclusions.

In conclusion, ultrasonic measurements such as DSH, DSE, DSV, HMD, and tongue width and thickness have a predictive value for difficult airway, and when the ultrasonic measurement of HMD is ˂5.29 cm, we should pay attention to the difficulty of laryngoscope exposure, and when DSE is ˂4.85 cm, watch out for difficult tracheal intubation. In terms of other ultrasound indexes, HMD is more valuable in predicting difficult airway.

## Figures and Tables

**Figure 1:** Ultrasonic images of each plane.

**Figure 2:** ROC curve of difficult laryngoscope exposure predicted by BMI, MMT, TMH, DSE, DSH, DSV, HMD, and tongue width and thickness.

**Figure 3:** The ROC curve of difficult laryngoscope exposure predicted by TMD and TMH.

**Figure 4:** ROC curve analysis of difficult tracheal intubation predicted by BMI, MMT, TMH, DSE, DSH, DSV, HMD, and tongue width and thickness.

**Figure 5:** ROC curve analysis of difficult tracheal intubation predicted by TMD and TMH.

**Table 1:** Comparison of the general conditions of patients in the four groups ($\bar{x}$_ _±_ _*s*).

Index	DL (*n* = 26)	NDL (*n* = 174)	*t*/*χ*^2^	*P*	DI (*n* = 17)	NDI (*n* = 183)	*t*/*χ*^2^	*P*
Gender (male/female)	15/11	89/85	0.388	>0.05	11/6	93/90	0.680	>0.05
Age (years)	50.15 ± 11.24	47.13 ± 14.41	1.022	>0.05	49.77 ± 12.43	47.31 ± 14.42	0.762	>>0.05
Height (cm)	168.67 ± 6.78	168.33 ± 7.25	0.225	>0.05	170.08 ± 6.92	168.62 ± 7.61	0.923	>0.05
Body weight (kg)	69.68 ± 11.94	63.35 ± 9.45	3.072	˂0.01	71.42 ± 10.12	63.75 ± 9.07	3.303	˂0.01
BMI (kg/m^2^)	24.36 ± 3.41	22.27 ± 2.36	3.949	˂0.01	24.57 ± 2.37	22.35 ± 2.58	3.415	˂0.01

**Table 2:** Comparison of the measurement indexes of the four groups of patients ($\bar{x}$_ _±_ _*s*).

Index	DL (*n* = 26)	NDL (*n* = 174)	*t*/*χ*^2^	*P*	DI (*n* = 17)	NDI (*n* = 183)	*t*/*χ*^2^	*P*
MMT (*n*/%)			63.225	˂0.01			79.309	˂0.01
I grade	5(19.23)	61(35.06)			5(29.41)	62(33.88)		
II grade	12(46.15)	113(64.94)			4(23.53)	120(65.57)		
III grade	9（34.62）	0（0.00）			8 (47.06)	1 (0.55)		
IID (cm)	4.31 ± 0.33	4.47 ± 0.36	2.135	˂0.05	4.62 ± 0.28	4.49 ± 0.38	1.375	>0.05
TMD (cm)	6.67 ± 0.51	6.91 ± 0.42	2.640	˂0.01	6.74 ± 0.51	6.93 ± 0.41	1.789	>0.05
ULBT (*n*/%)			0.396	>0.05			0.282	>0.05
I grade	14（53.85）	105（60.34）			9 (52.94)	109 (59.56)		
II grade	12（46.15）	69（39.66）			8 (47.06)	74 (40.44)		
TMH (cm)	4.76 ± 0.45	4.93 ± 0.28	2.636	˂0.01	4.72 ± 0.14	4.93 ± 0.25	3.409	˂0.01
DSE (cm)	1.85 ± 0.13	1.75 ± 0.14	3.427	˂0.01	1.91 ± 0.05	1.78 ± 0.14	3.799	˂0.01
DSH (cm)	0.96 ± 0.11	0.93 ± 0.12	1.201	>0.05	1.03 ± 0.15	0.92 ± 0.13	3.293	˂0.01
DSV (cm)	0.78 ± 0.05	0.75 ± 0.07	2.104	˂0.05	0.77 ± 0.04	0.73 ± 0.04	3.944	˂0.01
HMD (cm)	5.47 ± 0.22	5.63 ± 0.15	3.582	˂0.01	5.47 ± 0.23	5.66 ± 0.08	3.380	˂0.01
Tongue width (cm)	4.49 ± 0.13	4.36 ± 0.16	3.950	˂0.01	4.48 ± 0.13	4.36 ± 0.17	2.832	˂0.01
Tongue thickness (cm)	5.63 ± 0.15	5.47 ± 0.22	3.582	˂0.01	5.66 ± 0.08	5.47 ± 0.23	3.380	˂0.01

**Table 3:** Predictive efficacy of different indicators for difficult laryngoscope exposure.

Measurement index	Boundary value	Accuracy rate (%)	Sensitivity (%)	Specificity degree (%)	PPV (%)	NPV (%)	AUC
BMI	22.834 kg/m^2^	63.7	71.8	62.6	22.8	91.6	0.715
MMT	2 grade	41.6	81.3	35.4	16.2	92.3	0.797
ULBT	2 grade	58.6	47.5	60.4	15.4	88.3	0.533
TMD	6.52 cm	80.4	39.7	70.4	16.9	88.5	0.873
TMH	4.81 cm	67.1	71.8	66.5	24.8	93.7	0.741
IID	4.56 cm	51.2	79.4	46.8	18.6	93.5	0.737
DSE	1.78 cm	69.4	75.6	68.4	26.6	94.9	0.676
DSH	0.89 cm	51.8	71.6	48.3	17.6	91.7	0.662
DSV	0.75 cm	66.4	66.1	66.5	23.1	92.5	0.614
HMD	5.08 cm	60.3	88.6	55.7	23.6	97.3	0.812
Tongue width	4.36 cm	60.3	88.6	55.7	23.6	97.3	0.738
Tongue thickness	5.56 cm	69.4	75.6	68.4	26.6	94.9	0.776

**Table 4:** Comparison of the accuracy of ultrasonic indexes in predicting difficult laryngoscope exposure.

Measurement index	Exact number of cases	Inaccurate number of cases	Accuracy rate	*χ * ^2^	*P*
DSE	147	53	73.5	—	—
DSH	106	94	53.0	18.080	˂0.05
DSV	128	72	64.0	4.201	˂0.05
HMD	120	80	60.0	8.212	˂0.05
Tongue width	120	80	60.0	8.212	˂0.05
Tongue thickness	139	61	69.5	0.785	>0.05

Note: compared with DSE, ^*∗*^*P* < 0.05.

**Table 5:** Predictive efficiency of different indexes for difficult endotracheal intubation.

Measurement index	Boundary value	Accuracy rate (%)	Sensitivity (%)	Specificity degree (%)	PPV (%)	NPV (%)	AUC
BMI	23.083 kg/m^2^	67.1	75.9	66.3	16.9	96.7	0.751
MMT	2 grade	36.6	72.8	33.7	9.1	93.3	0.703
ULBT	2 grade	58.6	45.7	59.6	9.24	92.5	0.524
TMD	6.51 cm	60.5	97.3	56.8	16.6	99.4	0.801
TMH	4.79 cm	53.4	97.2	49.5	14.6	99.4	0.761
IID	4.62 cm	80.7	39.6	68.8	20.9	98.6	0.795
DSE	1.84 cm	49.1	84.7	45.9	12.4	97.2	0.668
DSH	0.87 cm	53.5	93.4	49.5	14.2	98.6	0.654
DSV	0.76 cm	72.6	69.6	72.7	18.8	96.5	0.663
HMD	5.08 cm	80.6	90.5	68.5	20.6	98.9	0.816
Tongue width	4.35 cm	53.4	97.2	49.5	14.6	99.4	0.761
Tongue thickness	5.50 cm	60.5	97.3	56.8	16.6	99.4	0.801

**Table 6:** Comparison of the accuracy of ultrasonic indexes in predicting difficult endotracheal intubation.

Measurement index	Exact number of cases	Inaccurate number of cases	Accuracy rate (%)	*χ * ^2^	*P*
DSE	163	37	81.5	—	—
DSH	106	94	53.0	36.880	˂0.01
DSV	145	55	72.5	4.573	˂0.05
HMD	107	93	53.5	35.738	˂0.01
Tongue width	107	93	53.5	35.738	˂0.01
Tongue thickness	121	79	60.5	21.418	˂0.01

Note: compared with DSE, ^#^*P* < 0.05.

## Data Availability

The datasets used and analyzed during the current study are available from the corresponding author upon reasonable request.
